The article "Influence of Good Death Perception, Moral Anguish, and End-of-life Care Attitude on End-of-life Care Performance of General Hospital Health Managers" was retracted in 2023. Reasons: unreliable results or conclusions; lack of ethics approval or compliance; concerns about the data; concerns about the peer review.

# Influence of Good Death Perception, Moral Anguish, and End-of-life Care Attitude on End-of-life Care Performance of General Hospital Health Managers

**DOI:** 10.1155/2022/7284959

**Published:** 2022-08-17

**Authors:** Min-Jung Lee, Nam-Joo Je

**Affiliations:** ^1^Graduate School of Nursing, Changshin University, Changwon, Republic of Korea; ^2^Department of Nursing, Changshin University, Changwon, Republic of Korea

## Abstract

This study attempted to identify the influence of good death perception, moral anguish, and End-of-life (EOL) care attitudes on the End-of-life (EOL) care performance of General Hospital Health Managers (GHHMs). This study was a quantitative and descriptive survey. The respondents of this study were 156 GHHMs working in three general hospitals with 300 beds or more and one general hospital with 100 beds or more in one of the cities in South Korea. The survey data were obtained from September 20 to October 20, 2021, and a total of 156 responses were analyzed by multiple linear regression using IBM SPSS/WIN 24.0 program. Results of the study revealed that it can be said that the higher the good death perception and the higher the moral anguish, the better the EOL care performance. The total explanatory power was 23.4%, and good death perception and moral distress explained EOL care performance by 23.4%. Furthermore, the general hospital managers' good health perception, moral anguish improved the performance and work satisfaction among nurses. It was necessary to implement a systematic EOL care education program to facilitate quality EOL care. Communication problems and lack of time are obstacles to EOL care performance, so hospital managers and the head of the nursing department provide communication-related education to EOL care GHHMs and allocate appropriate manpower so that GHHMs can actively and efficiently perform EOL care. It can be said that the higher the good death perception, the higher the moral anguish, and the higher the degree of EOL care performance. This study was meaningful in revealing good death perception, and moral agony in clinical practice have a significant effect on EOL care performance.

## 1. Introduction

General Hospital Health Managers (GHHMs) are in the immediate position to provide EOL care and counseling for patients and their families. EOL care constitutes an important part of palliative care, and it refers to the support and care given during the time surrounding death, which can be days, weeks, or even months [1]. GHHMs play a very important role as EOL care providers who can help patients safely accept death and prepare for death. IGHHMs must understand and learn how to recognize ethical problems, how to solve problems, and what actions to take in EOL care situations where ethical problems frequently occur.

Death is a natural phenomenon for humans. Some died in their homes with their families or relatives. According to the National Statistical Office [2], 74.9% of hospitals and 15.3% of families were on their deathbeds, and deaths in hospitals were much higher than those at home [2]. Recently, due to the changes in family structure, such as aging and nuclear familiarization, the number of people dying in medical institutions is increasing [3]. It can be inferred that as the place of death is moved from home to hospital, care and management for deathbeds change from family to medical institutions, and the proportion of deathbed nursing in nurses' work is increasing [4]. In addition, the majority of dying care and dying management of the elderly and chronically ill are transferred from families to various medical institutions and nurses [4]. However, research on EOL care has been conducted among nursing hospital nurses [5], hospice palliative care nurses [6], and a nurse who takes care of cancer patients [7], but studies on clinical nurses at university hospitals are limited [8]. Most of the study respondents were emergency room nurses who experienced death frequently, nurses on intensive care units, nursing hospital nurses who could prepare for death, and clinical nurses at relatively severe university hospitals. However, since most medical institutions, including general hospitals, operate mainly on disease treatment, EOL care is performed without sufficient education on EOL care. Performing EOL care without sufficient education on EOL care leads to anxiety about death when performing EOL care, and it is not possible to actively participate in EOL care via the negative death perception and attitude, so further research on EOL care by GHHMs is needed.

Do general hospital health managers' good death perception, moral anguish, and EOL care attitude affect GHHM's EOL Care Performance?

## 2. Theoretical Background

Recently, interest in EOL care based on human dignity has been growing, such as the implementation of the life-sustaining care decision system and the expansion of hospice and palliative care services. The more important the perception of a good death was, the more positive the EOL care attitude was, and most studies on good death perception were conducted on nursing students. Hospital workers often face death or EOL situations, and helping dying patients end their lives peacefully and reverently is increasingly emerging as one of the most important roles for hospital workers [7]. Nurses experience moral anguish in many moral issues that require ethical judgment in performing professional nursing and providing quality nursing care [9]. Regarding moral anguish, there have been studies that confirmed nursing hospitals and intensive care unit nurses, but studies on health managers in general hospitals are lacking, so it is necessary to study them. In addition, most EOL care performance studies confirmed the fragmentary relationship between EOL care performance, death perception, EOL care stress, and resilience. Studies on the integrative relationship between the two have been lacking.

Recently, as awareness of death and interest in good death perception increase, studies on good death perception are being attempted. In Korea, the term “good death” is unified, including both elements of “respectful death” and “comfortable death” [10]. Previous studies have reported that the perception of a good death among nurses affects their influencing EOL care [11]. Moral anguish refers to an uncomfortable and painful feeling and an experience when moral decisions have been made about how to do it. It cannot be moved into action [12]. Hospice and palliative care services are expanding under the Life-sustaining Treatment Decision Act, which took effect on April 7, 2020. Interest in death with dignity is increasing, and moral anguish is increasing in many moral dilemmas requiring ethical judgment skills in providing dying care for nurses [9].

“Death care attitude means positive or negative perceptions, emotions, and motivation of nurses for caring for terminally ill patients,” which is a major factor determining the overall health and quality of life of the deceased and their families [13]. Effective EOL care provides quality care to nonviable EOL patients and takes care of their families with love, allowing patients to live comfortably at dawn while maintaining dignity and dying without rejection [14].

Summarizing previous studies, end-of-life care performance had a positive correlation with awareness of good death [15] and attitudes toward end-of-life care [7]. Furthermore, awareness of good death [11] and attitudes toward end-of-life care [7] were meaningful factors that influenced end-of-life care performance.

EOL care is a holistic caring act that meets the physical, spiritual, social, and mental needs of the patient and his/her family, including those who are about to die. It has a broad meaning not only to provide nursing care for the rest of the life of the subject but also to reduce the pain of the patient at the end of his life and to comfortably meet the end of life while maintaining the quality and dignity of life for the rest of his life [16]. As for the performance of dying nursing by intensive care unit nurses, the positive death perception and dying nursing attitude, and the more death-related education they receive, the higher the EOL care performance [17]. Therefore, it can be seen that to improve the performance of EOL care by GHHMs, positive EOL care attitudes and good death awareness must be cultivated, and education on EOL care is necessary. However, most of the studies on the good death perception of clinical nurses and the performance of EOL care were conducted on nurses in elderly care facilities, cancer wards, and intensive care units. Therefore, there is a need for a study on the effect of good death perception, moral anguish, and EOL care attitude on the performance of the GHHMs towards patients in general hospitals.

## 3. Aim

This study was a descriptive study to understand the influencing factors of good death perception, moral anguish, and end-of-life nursing attitude of general hospital health managers on the performance of death-care nurses. This study attempted to identify the influence of good death perception, moral anguish, and EOL care attitudes on the EOL care performance of GHHMs and the development of EOL care programs for GHHMs.

### 3.1. Research Questions

- Do factors identified in previous studies, i.e., age, EOL education level, previous EOL care experience, EOL care attitude, etc. affect the EOL care performance of GHHMs?
- Are you influenced by your clinical experience in different healthcare settings?
- To what extent are GHHMs' death perceptions toward EOL care positive?
- Do perceptions of a good death, moral anguish, and EOL caring attitude affect the EOL caring performance of GHHMs?

## 4. Methods

### 4.1. Research Design

This study uses a quantitative approach in data collection and descriptive research study to understand the influence of good death perception, moral anguish, and EOL care attitudes on the EOL care performance of GHHMs.

### 4.2. Collection of Respondents of the Study, Data Collection, and Analysis Method

The research respondents of this study were 156 GHHMs working in three general hospitals with 300 beds or more and one general hospital with 100 beds or more in one of the cities in South Korea. The criteria for selecting the target are those who have worked for more than three months with dying patients, understood the purpose of the study, and voluntarily agreed to participate in it regardless of the working department.

The sampling size was calculated with a significance level (*α*) of .05 for regression analysis [18] using the G*∗*power 3.1.9.4 program, an effect size of .15 for power (1-*β*) .80, and 18 predictors. A total of 180 copies were distributed, and in consideration of the dropout rate of 20%, 174 copies were collected. Finally, 156 copies were used for data analysis, excluding 18 copies with insufficient or incomplete data.

The procedure of this study was approved by the Bioethics Committee (IRB) of University C (CSIRB-R2021041) after the preparation and deliberation of the research plan. For ethical consideration of this study, data collection was conducted from September 14 to October 15, 2021, after the IRB approval. For the survey, four general hospitals located in one of the cities in South Korea were randomly sampled. The purpose of the study was explained to the head of the institution and the head of the nursing department by e-mail or telephone, and cooperation was sought. The research purpose, research method, and participation method were explained to the target respondents. Finally, the research was conducted among the GHHMs after obtaining their approval and voluntary participation in the study.

After gaining the respondents' consent, a total of 180 questionnaires were distributed and only 174 were recovered. It took about 15 to 20 minutes to fill out the questionnaire. Excluding the 18 responses with insufficient or incomplete data, 156 completed surveys were used for data analysis.

After data analysis using IBM SPSS/25 statistical program, the significance level of the results was 0.05. For general characteristics, the frequency (percentage), mean, and standard deviation were calculated for the values of each item. Differences in perception of a good death, moral pain, EOL care attitude, and EOL care performance according to the general characteristics of respondents were measured by *t*-test for two groups and one-way ANOVA for three or more groups to know the correlation between the independent variable and the dependent variable. The analysis was performed using Pearson's correlation coefficient. To find out the factors affecting the dependent variable, hierarchical multiple regression analysis was used to identify the factors affecting the EOL care performance, which is the dependent variable.

### 4.3. Research Instruments

The research instruments used in this study have 104 questions consisting of 15 questions for the subject's general characteristics, 17 questions for good death perception, 21 questions for moral anguish, 30 questions for EOL care attitude, and 22 questions for EOL care performance. Each research instrument received prior permission from the author through e-mail and paid-for tools that required tool usage fees. The research instruments whose validity has been verified in previous studies were used.

#### 4.3.1. General Characteristic

The general characteristics of the respondents were measured with a total of 15 questions [19], including age, gender, family type, education level, total work experience, current work experience, work type, job satisfaction, work satisfaction, religion, religious influence, number of meaningful people's death experiences, death-related education, and EOL care experience. The criteria for selection of study respondents are those who have worked with the dying patient for more than 3 months.

#### 4.3.2. Good Death Perception

The good death perception was measured using the Korean version of「The concept of a good death scale」developed by Schwartz et al. [20] for medical students, nursing students, graduate students in life science, and nurses in hospice nursing activities. It has a total of 17 questions divided into three subareas, namely: clinical symptoms (5 questions), which focus on the clinical or biomedical aspects of the death process; intimacy (9 questions), which is related to the psychosocial and spiritual aspects of the death process; and, sense of control (3 questions), which is the ability to control consciousness, communication, and physical function in the process of death. Each item was rated using a four-point Likert scale ranging from “not important at all (1 point)” to “very important (4 points).” The higher the score, the higher the perception of a good death. In the study of Schwartz et al. [20], the reliability of the tool was Cronbach's *α* .87 and in this study, it was Cronbach's *α* .80.

#### 4.3.3. Moral Anguish

Moral anguish was measured using「Moral Distress Scale for Psychiatric Nurses: MDS-P」by Ohnishi et al. [21] with 21 items adapted, revised, and supplemented by Noh et al. [12]. Each item was rated using a seven-point Likert scale ranging from “experienced but not at all uncomfortable (0 points)” to “very uncomfortable (6 points)” according to the degree of experience of uncomfortable and negative emotions about moral distress situations. The higher the score, the greater the moral anguish. At the time of tool development, the reliability was Cronbach's *α* 0.90, in the study of Noh et al. [22], it was 0.83, and in this study, it was 0.95.

#### 4.3.4. EOL Care Attitude

The EOL care attitudes were measured using the the「Attitudes toward Nursing Care of the Dying Scale」tool developed by Frommelt [23] and modified and supplemented by Cho and Kim [24]. This tool consists of 30 questions in three subareas: EOL awareness (9 items), EOL emotion (6 items), and EOL care (15 items). Each item was rated using a four-point Likert scale ranging from not (1 point) to “strongly agree” (4 points), and negative questions were converted inversely. Scores ranged from 30 to 120 points. The higher the score, the more positive the EOL care attitude. At the time of tool development, the reliability was Cronbach's *α* = .94, in the study of Cho and Kim [24]; it was .86, and in this study, it was .78.

#### 4.3.5. EOL Care Performance

The EOL care performance was measured using the tool developed by Park and Choi [25]. This tool consists of 22 items in three subareas: physical area (8 items), psychological area (8 items), and spiritual area (6 items). Each item is rated on a four-point Likert scale ranging from not at all (1 point) to “always” (4 points). Scores ranged from 22 to 88, with higher scores indicating higher EOL care performance. In the study of Park and Choi [25], the reliability of the tool was Cronbach's *α* .93, and in this study, it was .92.

### 4.4. Ethical Considerations

The selection process of the respondents and the purpose of the study were explained to the head of the institution and the head of the nursing department of the four general hospitals. After gaining their approval, the research purpose, the rights of research participants, and the research (e.g., confidentiality and anonymity) were explained to the nurses. Those who voluntarily participated were distributed with the questionnaires. The completed questionnaires were stored and encrypted for safety. The data will be kept for three years after the end of the study. Then these will be shredded. A copy of the consent form was provided to the respondents, and the respondents who responded to the survey were returned with a small gift.

## 5. Results

### 5.1. General Characteristics of Respondents

In the general characteristics of the respondents, the average age of the participants was 37.58 ± 10.22 years, and 52 people (33.3%) were the most under 29 years old. As for gender, there were 150 women (96.2%). A total of 86 persons (55.1%) were married. The number of college graduates and university graduates was equal to 78 (50%) responses. The average clinical experience was 9.62 ± 7.48 years, and those with less than five years had the most with 52 (33.3%) respondents. The average current hospital experience was 6.58 ± 6.20 years, and 48 patients (30.8%) had less than three years. The most common type of work was three shifts with 112 (71.8%) people. As for job satisfaction, 90 (57.7%) people were most satisfied, and 81 (51.9%) people were satisfied with their job. Regarding the presence or absence of religion, 83 (53.2%) people answered that they have religion, and the degree of influence of religion had no effect with 68 (43.6%) people. A total of 116 (74.4%) people said that they had no experience of death that of family/acquaintances within one year. No experience of EOL education was the most at 83 (53.2%) responses. In the case of 73 people with educational experience, the most common education route was continuing education with 33 (45.2%) people. The average monthly number (more than five months) of nursing care for EOL patients had 123 (78.8%) responses (Table 1).

### 5.2. Subject's Good Death Perception, Moral Anguish, EOL Care Attitude, and EOL Care Performance

Good death perception was 49.57 ± 5.67 points (out of 68 points), and the average score was 2.92 ± 0.33 points (out of 4 points). Moral anguish was 80.65 ± 18.49 points (126 points), and the average score was 3.85 ± 0.88 points (out of 6 points). The EOL care attitude was 85.64 ± 6.79 points (out of 108 points), and the average score was 2.85 ± 0.23 points (out of 4 points). EOL care performance was 59.27 ± 10.01 points (out of 88 points), and the average score was 2.69 ± 0.45 points (out of 4 points) (Table 2).

### 5.3. Differences in Good Death Perception, Moral Anguish, EOL Care Attitude, and EOL Care Performance according to Subject's General Characteristics

Significant differences in the perception of a good death were found in job satisfaction (*F* = 7.92, *p*=0.001), work satisfaction (*F* = 3.89, *p*=0.039), and the average monthly number of nursing care for dying patients (*t* = 2.20, *p*=0.029). There were also differences in moral anguish in the last educational background (*t* = −1.99, *p*=0.049), clinical experience (*F* = 4.85, *p*=0.003), and the average monthly number of nursing care for dying patients (*t* = −2.19, *p*=0.030). The characteristics that showed differences in EOL care attitude were final educational background (*t* = −3.82, *p* < 0.001), EOL education experience (*t* = 3.93, *p* < 0.001), and average monthly number of EOL care (*t* = -2.87, *p*=0.005). The characteristics that showed differences in EOL care performance were job satisfaction (*F* = 4.97, *p*=0.008), work satisfaction (*F* = 10.14, *p* < 0.001), religious status (*t* = −2.91, *p*=0.004), and religion (*F* = 7.36, *p*=0.001) [Table 3].

### 5.4. The Relationship between Good Death Perception, Moral Anguish, EOL Care Attitude, and EOL Care Performance

There was a positive correlation between good death perception (*r* = .29, *p* < 0.001), moral anguish (*r* = .19, *p*=0.016), and EOL care attitude (*r* = .17, *p*=0.029) (Table 4).

### 5.5. Factors Affecting EOL Care Performance

Multiple regression analysis using a hierarchical selection method was performed to test factors affecting EOL care performance, and the results are shown in Table 5. Among the characteristics of the respondents, job satisfaction (dissatisfaction criteria), religious presence (no criteria), and degree of influence of religion (does not affect criteria), which showed a significant difference in EOL care performance, were input into Model 1. The general characteristics were treated as dummy variables. In Model 2, in addition to Model 1, good death perception, moral anguish, and EOL care attitude were added. Job satisfaction was excluded from the analysis as it showed a high correlation with work satisfaction. As a result of checking whether there is a correlation between the error terms before analysis, the Durbin-Watson statistic was 1.91, which is a value near 2, so there was no correlation between the error terms. As a result of examining whether the distribution of error terms can be assumed to be normal through standardized residuals, all values are within ± 3, so the distribution of error terms can be assumed to be normal. As a result of examining whether there is multicollinearity between the input independent variables through the tolerance limit and the variance expansion factor, the tolerance limit was .26 to .93, which was more than .10, and the variance expansion factor was 1.08 to 3.78, showing a value less than 10. There was no multicollinearity between them. Among the characteristics input in Model 1, the variables that had a significant effect on EOL care performance were “satisfaction” (*β* = .39, *p*=0.007) of work satisfaction and “affected” on the degree of religious influence (*β* = .23, *p*=0.023). In other words, it can be said that the more satisfied the work satisfaction compared to the dissatisfaction, the better the EOL care performance is. The explanatory power by Model 1 was 17.3% (*F* = 6.29, *p* < 0.001, *R*^2^ = .173, Adj-R^2^ = .146). In Model 2, the variables that had a significant effect on work satisfaction were “satisfaction” (*β* = .38, *p*=0.007), and the degree of religious influence was “affected” (*β* = .20, *p*=0.038). Additionally, good death perception (*β* = .22, *p*=0.003) and moral anguish (*β* = .16, *p*=0.040) were found to have a significant effect on EOL care performance. However, EOL care attitude (*β* = .12, *p*=0.131) did not have a significant effect. In other words, it can be said that the higher the good death perception, the higher the moral anguish, and the higher the degree of EOL care performance. The proportion additionally explained by Model 2 was 10.0%, and the total explanatory power of Model 2 was 23.4% (*F* = 6.92, *p* < 0.001, *R*^2^ = .273, Adj- *R*^2^ = .234) (Table 5).

## 6. Discussion

The purpose of this study is to identify the influence of good death perception, moral anguish, and EOL care attitudes on the EOL care performance of GHHMs. An attempt was made to provide basic data, and based on the results of this study, we would like to discuss it as follows.

### 6.1. Good Death Perception, Moral Anguish, And EOL Care Attitude of GHHMs Performing EOL Care

The good death recognition score of this study subject was higher than the average. Kim and Kim [8] study's, which used the same tools for clinical nurses, also showed good death recognition scores similar to this study. Using the same tools, the results of Bang's (2018)'s study on nursing hospital nurses and Jo and Ki's (2021)'s research on university hospital nurses were also similar. This seems to have resulted in similar results because the environmental similarity of a nurse currently working in the hospital field, the perception of death, and ethical consciousness are socially recognized concepts rather than individual values. Because good death perception is interpreted differently by each individual through socialization under specific social, cultural, and historical environments [26], it is very important to understand the good death perception of GHHMs who care for patients about to die. Unlike nursing hospitals and hospice wards, GHHMs deal with a variety of EOL patients. Therefore, when performing EOL nursing, care is needed to help the patient reflect on the value of his or her life and organize their thoughts. It is necessary to raise a positive attitude toward death among GHHMs so that they can prepare for the EOL care performance of patients nearing death.

As a result of this study, the degree of moral anguish of GHHMs was higher than the average, which was rather positive. The results of this study were reported by Noh et al. [22] similar to the results of a study on the moral anguish of nurses caring for mentally ill patients using the same tools as in this study. However, the results were higher than those of Son [26], who studied the moral anguish of emergency room nurses. This is a study to understand the effect of the ethical environment of the emergency room on moral anguish. Nurses working in the emergency room are considered to have a relatively low moral anguish score due to the inadequacy of the intervention role of nurses due to the high influence of the direct involvement of doctors because of the characteristics of their work. In the future, through advanced, in-depth interviews on the moral anguish of nurses working in various types of institutions, a study to compare the differences between the moral anguish experiences that may occur between regions, medical systems, and differences in bed size should also be conducted. In addition, it is necessary to develop a protocol to cope well with moral anguish in the future, and for this, it is necessary to study various cases in depth. The goal of end-of-life care is to prevent or relieve suffering as much as possible while respecting the desires of dying patients. Open communication and shared decision-making among health care providers, patients, and families would avoid many of the ethical dilemmas in end-of-life care [27].

In this study, the EOL caring attitude was higher than the average. It was similar to Choi's [28] EOL care attitude toward cancer center nurses. In a study conducted by Hwang [29] with nurses in the internal medicine ward, the score was higher than in this study. EOL care attitude refers to the positive or negative attitudes nurses have toward caring for terminally ill patients. The more positive a nurse's EOL care attitude is, the better quality care can be provided to EOL patients [20]. A positive EOL care attitude positively affected the EOL care attitude of general hospital nurses based on the study [18] that a positive EOL care attitude lowered the desire to avoid the dying patient and the fear of death, and could more actively perform EOL care. As a result of this study, GHHMs have relatively few opportunities and benefit from systematic EOL care education. Therefore, multifaceted efforts are needed to positively change EOL care attitudes through EOL care education.

In this study, the average degree of GHHM's EOL care performance was higher than the average. The score of the EOL caring performance subitem was highest in the psychological domain, high in the physical domain, but the lowest in the spiritual domain. The results of this study were similar to the average of Ko and Moon [17], who studied factors affecting the EOL care performance of nursing home caregivers using the same tools as in this study. The score of the EOL care performance subitem was highest in the physical domain, followed by the psychological domain, and the lowest in the spiritual domain. Comparing the study results, both the GHHMs and nursing hospital nurses performed EOL care performance above average. Nursing performance was the highest. In addition, they both showed low nursing performance in the spiritual realm, indicating that most of them focused on physical and psychological nursing. It can be inferred that spiritual nursing is insufficient due to communication problems and lack of time. Based on the previous research and the results of this study, it suggests that there is a need for program development and reinforcement education that can strengthen the spiritual realm when performing EOL care.

### 6.2. Good Death Perception, Moral Anguish, EOL Care Attitude, and EOL Care Performance according to General Characteristics of GHHMs

As a result of examining the difference in the degree of EOL care performance according to the general characteristics of general hospital nurses, there were significant differences according to the degree of influence of religion, the experience of the death of family/acquaintances within 1 year, the experience of EOL education, education route, and an average number of nursing care for EOL patients. This is similar to the study of Han and Choi [30], where there is a significant difference in the degree of role performance according to age, marital status, educational background, and status which were found to be high and consistent with this study. It is thought that EOL care performance may have increased as the understanding of EOL patients increased due to the increase in competency according to clinical experience. Therefore, in clinical practice, it is necessary to allocate and adjust the manpower of specialized hospice nurses so that EOL patients can receive proper care by placing them as nurses with experience in EOL care. In this study, the result that the degree of EOL care performance was higher in patients with more than 15 years of clinical experience than those with more than 5 to 10 years of clinical experience was similar to that of Noh et al. [7], who studied nurses caring for cancer patients. It is thought that the performance of EOL care was improved as the practical ability was allowed to improve as time went by, and the understanding of the dying patient was increased due to the increase in competency according to the clinical experience. In this study, the job satisfaction of GHHMs was higher in “satisfaction” than “dissatisfied” or “normal.” Although it is difficult to make a comparison because there is no direct study on EOL care performance and job satisfaction, the results of examining the relationship between nursing job satisfaction and nursing job performance for nurses were similar to those of Son and Park [31] for clinical nurses. In this study, the job satisfaction of nurses in general hospitals was statistically significant in the nurses' EOL care performance. It can be said that the more satisfactory the work satisfaction compared to the dissatisfaction, the better the EOL care performance. The degree of EOL care performance was higher in “satisfaction” than “dissatisfied” or “average” in nursing work, and “satisfaction” in general hospital work than “dissatisfied” or “normal.” These results can be seen as having a positive and active work attitude toward EOL care performance and satisfaction with the nursing work of caring for patients with professional knowledge and judgment. In a study by Son and Park [31] targeting clinical nurses, EOL care performance showed a significant difference depending on nursing job satisfaction and EOL care education experience.

### 6.3. Effect of Good Death Perception, Moral Anguish, and EOL Care Attitudes on EOL Care Performance

As for influencing factors on EOL care performance in this study, it can be said that the degree of EOL care performance is higher as job satisfaction is more satisfactory than dissatisfaction, the degree of religious influence has an effect, and good death perception and moral anguish are higher. In a study by Kim et al. [11] targeting general hospital nurses, in the order of good death perception, education experience related to life-sustaining treatment, the stress in nursing care for life-sustaining treatment, and knowledge of advance directives for life-sustaining treatment, EOL care stress was the most influencing factor in the study of Ko and Moon [17], targeting intensive care nurses, and in the order of medical personnel and EOL care attitude, which are subdomains of EOL care obstacle factors. Unlike previous studies, in this study, new variables such as job satisfaction, religion, and moral anguish were identified as variables affecting EOL care performance. In the future, it is necessary to check the explanatory power through repeated studies, including the variables of the previous study and the variables of this study.

To positively change EOL care performance, it is necessary to raise the awareness of the good death and to change the perception of death by preparing and intervening in a well-dying (good death) education program for those in medical institutions such as hospitals. The degree of EOL care performance was higher as the total hospital work experience increased, which was similar to the study of Son and Park [31] and the study of emergency room nurses by Son [26]. It is thought that there is a need for an educational program to positively raise awareness of death through the education of nurses. The more specialized knowledge and skills there are, the fewer difficulties in performing EOL care work, so it is thought that systematic education is necessary. Basic knowledge from undergraduate training and continuous training to develop clinical competence is a prerequisite for enabling GHHMs to provide high-quality EOL care [32]. The dying patients should not only focus on physical care but also provide psychological and spiritual care. To achieve this, it is considered necessary to develop a systematic nursing program. In this study, it is thought that the higher the professional knowledge and skills in EOL care, the fewer difficulties in performing EOL care work. Therefore, it is necessary to implement a systematic EOL care education program to facilitate quality EOL care. Communication problems and lack of time are obstacles to EOL care performance, so hospital managers and the head of the nursing department provide communication-related education to EOL care GHHMs and allocate appropriate manpower so that GHHMs can actively and efficiently perform EOL care. This study is significant in that it provided the basic information necessary for the development of end-of-life care programs for GHHMs by identifying the relationship between perceptions of a good death, moral anguish, and attitudes toward death and performance. GHHMs' good death perception and moral anguish affected EOL care performance. It can be said that the higher the good death perception, the higher the moral anguish, and the higher the degree of EOL care performance.

## 7. Conclusion

Good death perception and moral anguish were correlated, and EOL care attitude did not show a correlation with EOL care performance. Therefore, good death perception and moral agony in clinical practice have a significant effect on EOL care performance. In addition to this variable, it is considered that it is necessary to give active and continuous interest and administrative support along with efforts to identify other variables that explain EOL care performance. Furthermore, the results imply that there is a need for greater emphasis on further continuing education within EOL care for GHHMs working in all types of clinical specialties to encourage GHHMs to talk about death and to enhance attitudes toward EOL care. Since this study was conducted for some general hospitals, there are limitations in generalizing the study.

## 8. Recommendations

Based on the results of this study, we would like to make the following suggestions.

First, an in-depth study including variables other than good death perception and moral anguish is suggested to investigate the effect on EOL care performance. Second, based on the influencing factors of EOL care performance, we propose an experimental study to develop an intervention program to increase good death perception and reduce moral anguish, and verify the clinical application effect. Third, research on the development and application of tools applied to nursing assistants and caregivers is suggested.

## Figures and Tables

**Table 1:** General characteristics (*n* = 156).

Characteristics	Categories	*n* (%)	M ± SD
Age (yr)	≤23∼〉30	52 (33.3)	37.58 ± 10.22
	≤30∼〉40	39 (25.0)	
	≤40∼〉50	41 (26.3)	
	≤50∼≥65	24 (15.4)	
Gender	Male	6 (3.8)	
	Female	150 (96.2)	
Marriage	Single	70 (44.9)	
	Married	86 (55.1)	
Last educational background	College	78 (50.0)	
	University	78 (50.0)	
Clinical experience (years)	〉5	52 (33.3)	9.62 ± 7.48
	≤5∼〉10	39 (25.0)	
	≤10∼〉15	26 (16.7)	
	≤15	39 (25.0)	
Current hospital experience (years)	〉3	48 (30.8)	6.58 ± 6.20
	≤3∼〉5	31 (19.9)	
	≤5∼〉10	39 (25.0)	
	≤10	38 (24.3)	
Work type	Shift work	112 (71.8)	
	Dedicated to D/E/N	24 (15.4)	
	Day work	20 (12.8)	
Job satisfaction	Satisfaction	90 (57.7)	
	Moderate	58 (37.2)	
	Dissatisfaction	8 (5.1)	
Work satisfaction	Satisfaction	81 (51.9)	
	Moderate	62 (39.8)	
	Dissatisfaction	13 (8.3)	
Religion	No	73 (46.8)	
	Yes	83 (53.2)	
Degree of influence of religion	Affect	45 (28.8)	
	Usually	43 (27.6)	
	Does not affect	68 (43.6)	
Family/acquaintance death experience within 1 year	Yes	40 (25.6)	
	No	116 (74.4)	
EOL education experience	Yes	73 (46.8)	
	No	83 (53.2)	
Education path	Undergraduate class	12 (16.4)	
	Graduate class	4 (5.4)	
	Continuing education	33 (45.2)	
	Job training in hospitals/Other	23 (31.4)/1 (1.6)	
The average number of EOL care per month (times)	〉5	123 (78.8)	
	≤5	33 (21.2)	

**Table 2:** Subject's good death perception, moral anguish, EOL care attitudes, and EOL care performance (*n* = 156).

Variables	Range	Min	Max	Mean ± SD
Good death perception	17–68	34	68	2.92 ± 0.33
Moral anguish	0–126	16	126	3.85 ± 0.88
EOL care attitudes	30–120	73	108	2.85 ± 0.23
EOL care performance	22–88	37	88	2.69 ± 0.45

**Table 3:** Subject's good death perception, moral anguish, EOL care attitudes, and EOL care performance according to the general characteristics of the subject (*n* = 156).

Characteristics	Categories	Good death perception			Moral anguish			EOL care attitudes			EOL care performance		
		Mean ± SD	t/F	*P* (Scheffe)	Mean ± SD	t/F	*P* (Scheffe)	Mean ± SD	t/F	*P* (Scheffe)	Mean ± SD	t/F	*P* (Scheffe)
Age (yr)	≤23∼〉30	2.92 ± 0.33	1.04	0.376	3.61 ± 0.80	2.36	0.074	2.86 ± 0.24	1.52	0.213	2.65 ± 0.44	2.57	0.056
	≤30∼〉40	2.84 ± 0.35			3.85 ± 0.82			2.80 ± 0.20			2.57 ± 0.41		
	≤40∼〉50	2.96 ± 0.36			4.07 ± 1.01			2.90 ± 0.25			2.79 ± 0.48		
	≤50∼≥65	2.96 ± 0.26			3.99 ± 0.83			2.85 ± 0.19			2.83 ± 0.46		
Gender	Male	2.84 ± 0.23	−0.55	0.582	3.99 ± 0.95	0.40	0.689	2.87 ± 0.22	0.12	0.905	2.58 ± 0.43	−0.65	0.517
	Female	2.92 ± 0.34			3.84 ± 0.88			2.85 ± 0.23			2.70 ± 0.46		
Marriage	Single	2.91 ± 0.33	−0.03	0.978	3.72 ± 0.84	−1.74	0.084	2.88 ± 0.24	1.45	0.150	2.69 ± 0.51	−0.09	0.928
	married	2.92 ± 0.34			3.96 ± 0.91			2.83 ± 0.21			2.70 ± 0.41		
Last educational background	College	2.94 ± 0.36	0.75	0.456	3.71 ± 0.86	−1.99	0.049	2.79 ± 0.18	−3.82	<0.001	2.71 ± 0.46	0.43	0.662
	University	2.90 ± 0.31			3.99 ± 0.88			2.92 ± 0.25			2.68 ± 0.45		
Clinical experience (years)	〉5	2.94 ± 0.33	0.97	0.408	3.58 ± 0.89	4.85	0.003	2.85 ± 0.24	2.56	0.057	2.70 ± 0.49	0.22	0.885
	≤5∼〉10	2.86 ± 0.33			3.96 ± 0.89		d > a	2.85 ± 0.21			2.72 ± 0.41		
	≤10∼〉15	2.87 ± 0.37			3.68 ± 0.86			2.77 ± 0.19			2.63 ± 0.52		
	≤15	2.97 ± 0.32			4.22 ± 0.74			2.92 ± 0.23			2.70 ± 0.42		
Current hospital experience (years)	〉3	2.96 ± 0.33	1.61	0.188	3.65 ± 0.95	2.15	0.097	2.85 ± 0.22	0.40	0.761	2.61 ± 0.49	2.06	0.107
	≤3∼〉5	2.93 ± 0.32			3.72 ± 0.69			2.84 ± 0.24			2.86 ± 0.38		
	≤5∼〉10	2.82 ± 0.35			3.97 ± 0.87			2.84 ± 0.20			2.68 ± 0.47		
	≤10	2.95 ± 0.33			4.08 ± 0.90			2.89 ± 0.25			2.68 ± 0.42		
Work type	Shift work	2.91 ± 0.31	0.25	0.780	3.77 ± 0.90	1.60	0.205	2.85 ± 0.24	1.53	0.219	2.69 ± 0.48	0.06	0.942
	Dedicated to D/E/N	2.96 ± 0.37			4.00 ± 0.86			2.83 ± 0.17			2.71 ± 0.45		
	Day work	2.91 ± 0.40			4.10 ± 0.76			2.94 ± 0.18			2.67 ± 0.34		
Job satisfaction	Satisfaction	3.00 ± 0.33	7.92	0.001	3.88 ± 0.79	1.91	0.151	2.85 ± 0.21	0.41	0.665	2.79 ± 0.43	4.97	0.008
	Moderate	2.80 ± 0.30		a > b, c	3.73 ± 0.98			2.85 ± 0.23			2.56 ± 0.45		a > b,c
	Dissatisfaction	2.81 ± 0.40			4.35 ± 1.02			2.93 ± 0.32			2.58 ± 0.52		
Work satisfaction	Satisfaction	2.99 ± 0.34	3.89	0.023	3.81 ± 0.83	0.16	0.853	2.85 ± 0.23	0.82	0.443	2.84 ± 0.41	10.14	<0.001
	Moderate	2.84 ± 0.30		a > b	3.89 ± 0.93			2.84 ± 0.21			2.57 ± 0.44		a > c
	Dissatisfaction	2.86 ± 0.38			3.88 ± 1.02			2.93 ± 0.28			2.39 ± 0.49		
Religion	No	2.88 ± 0.29	−1.24	0.218	3.91 ± 0.91	0.81	0.419	2.87 ± 0.23	0.98	0.330	2.58 ± 0.47	−2.91	0.004
	Yes	2.95 ± 0.37			3.80 ± 0.85			2.84 ± 0.22			2.79 ± 0.42		
Degree of influence of religion	Affect	2.90 ± 0.35	1.49	0.238	3.87 ± 1.00	0.04	0.960	2.91 ± 0.25	2.22	0.113	2.87 ± 0.45	7.36	0.001
	Moderate	2.99 ± 0.37			3.82 ± 0.79			2.81 ± 0.24			2.73 ± 0.42		a > c
	Does not affect	2.88 ± 0.29			3.86 ± 0.87			2.85 ± 0.19			2.55 ± 0.44		
Family/acquaintance death experience within one year	Yes	2.89 ± 0.36	−0.64	0.524	4.03 ± 0.87	1.51	0.133	2.91 ± 0.25	1.85	0.066	2.72 ± 0.41	0.42	0.675
	No	2.93 ± 0.33			3.79 ± 0.88			2.84 ± 0.22			2.69 ± 0.47		
EOL education experience	Yes	2.97 ± 0.38	1.84	0.068	3.92 ± 0.95	0.99	0.322	2.93 ± 0.26	3.93	<0.001	2.76 ± 0.43	1.69	0.093
	No	2.87 ± 0.28			3.78 ± 0.82			2.79 ± 0.17			2.64 ± 0.47		
The average number of EOL care per month (times)	〉5	2.95 ± 0.31	2.20	0.029	3.77 ± 0.83	−2.19	0.030	2.83 ± 0.20	−2.87	0.005	2.68 ± 0.45	−0.98	0.329
	≤5	2.80 ± 0.40			4.14 ± 1.01			2.95 ± 0.28			2.76 ± 0.46		

**Table 4:** Correlation between good death perception, moral anguish, EOL care attitudes, and EOL care performance (*n* = 156).

	Good death perception	Moral anguish	EOL care attitudes	EOL care performance
	*r* (*p*)			
Good death perception	1			
Moral anguish	0.04 (0.634)	1		
EOL care attitudes	0.01 (0.890)	0.36 (<0.001)^∗^	1	
EOL care performance	0.29 (<0.001)^∗^	0.19 (0.016)	0.18 (0.029)	1

^∗^ *p* < 0.001.

**Table 5:** Multiple regression analysis on EOL care performance (*n* = 156).

	Model 1					Model 2				
	B	SE	*β*	*t*	*p*	B	SE	*β*	*t*	*p*
(Constant)	2.30	0.15		15.75	<0.001	0.43	0.53		0.82	0.415

*Work Satisfaction (Dissatisfaction Criteria)*										
Satisfaction	0.35	0.13	0.39	2.73	0.007	0.34	0.12	0.38	2.76	0.007

*Degree of influence of religion (Does not affect Criteria)*										
Affect	0.23	0.10	0.23	2.31	0.023	0.20	0.10	0.20	2.10	0.038
Good death perception						0.30	0.10	0.22	2.99	0.003
Moral anguish						0.08	0.04	0.16	2.08	0.040
Adj-R^2^	0.146					0.234				
*R * ^2^	0.173					0.273				
R^2^change amount	—					0.100				
F (*p*)	6.29 (<0.001)					6.92 (<0.001)				
F change amount (*p*)	—					6.75 (<0.001)				

Durbin-Watson = 1.91, Tolerance = .26∼.93, VIF = 1.08∼3.78. Dummy Variable = Work Satisfaction (Dissatisfaction 0), Degree of influence of religion (Does not affect 0).

## Data Availability

No data is available.

## References

[1] National Board of Health and Welfare (2016). *National Guidelines: Palliative Care 2016*.

[2] Statistics Korea (2016). A press release on the cause of death statistics in 2015. https://kostat.go.kr/portal/korea/kor_nw/1/6/2/index.board?bmode=read&bSeq=&aSeq=356345&pageNo=1&rowNum=10&navCount=10&currPg=&searchInfo=&sTarget=title&sTxt=.

[3] Woo Y. W., Kim K. H., Kim K. S. (2013). Death anxiety and terminal care stress among nurses and the relationship to terminal care performance. *The Korean Journal of Hospice and Palliative Care*.

[4] Kim W. S., Cho H. H., Kwon S. H. (2016). The influence of terminal care performance, death anxiety, and self-esteem on terminal care stress of geriatric hospital nurses. *The Korean Journal of Hospice and Palliative Care*.

[5] Sung B. M. (2018). Influence of Nursing Professionalism and Good Death Awareness on Terminal Care Attitude in Geriatrics Hospital Nurses.

[6] Cho E. J. (2019). Effects of nursing workplace spirituality, end-of-life care stress, and resilience on compassion fatigue in nurses of hospice and palliative care institutions.

[7] Noh S. S., Lee C. K., Sung Y. H. (2016). Predictors of terminal care performance of clinical nurses for cancer patients. *Journal of Korean Critical Care Nursing*.

[8] An H. N., Kim I. O. (2020). Factors affecting college students’ sexual autonomy. *Health & Nursing*.

[9] Lee J. S., Ahn S. H. (2019). The impact of moral sensitivity and moral distress on end-of-life care performance among intensive care unit nurses. *Korean Journal of Medical Ethics*.

[10] Kim M. S. (2015). Influence of moral sensitivity and ethical values on biomedical ethics awareness of nursing students. *The Journal of Korean Academic Society of Nursing Education*.

[11] Kim S. K., Kim S. H., Yun H. Y. (2019). Factors that influence end-of-life care provided by nurses in general hospitals. *Korean Journal of Medical Ethics*.

[12] Morley G., Ives J., Bradbury-Jones C., Irvine F. (2019). What is moral distress? A narrative synthesis of the literature. *Nursing Ethics*.

[13] Yang S. A. (2015). Convergence analysis of the factors influencing terminal care attitude. *Journal of the Korea Convergence Society*.

[14] Jo K. H., Park A. R., Lee J. J., Choi S. J. (2015). The effect of suffering experience, empathy ability, caring behaviors on terminal care performance of clinical nurses. *The Korean Journal of Hospice and Palliative Care*.

[15] Song E. H., Lee H. K. (2019). Effects of good death awareness and spiritual well-being on the elderly nursing performance of geriatric hospital nursing providers. *J Korean Appl Sci Technol*.

[16] National Health Service (2012). *End of Life Care*.

[17] Ko M. J., Moon S. H. (2016). Factors influencing performance of end-of-life care by ICU nurses. *Journal of Korean Academy of Psychiatric and Mental Health Nursing*.

[18] Fristedt S., Grynne A., Melin-Johansson C., Henoch I., Hagelin C. L., Browall M. (2021). Registered nurses and undergraduate nursing students’ attitudes to performing end-of-life care. *Nurse Education Today*.

[19] I’m P. Y. (2021). Effects of spirituality and terminal care attitude on the terminal care performance of nurses working in nursing hospital.

[20] Schwartz C. E., Mazor K., Rogers J., Ma Y., Reed G. (2003). Validation of a new measure of the concept of a good death. *Journal of Palliative Medicine*.

[21] Ohnishi S., Miyoshi T., Shirai S. (2010). Low temperature stress at different flower developmental stages affects pollen development, pollination, and pod set in soybean. *Environmental and Experimental Botany*.

[22] Noh D. B., Kim S. A., Kim S. H. (2013). Moral distress, moral sensitivity and ethical climate of nurses working in psychiatric wards. *Journal of Korean Academy of Psychiatric and Mental Health Nursing*.

[23] Frommelt K. H. M. (1991). The effects of death education on nurses’ attitudes toward caring for terminally ill persons and their families. *American Journal of Hospice and Palliative Medicine*.

[24] Cho H. J., Kim E. S. (2005). The effect of the death education program on the death anxiety and attitudes toward nursing care of the dying patients of nursing student. *Korean Journal of Hospice and Palliative Care*.

[25] Park S. J., Choi S. H. (1996). A study on the degrees of death orientation and terminal care performance of nurses. *Journal of Korean Academy of Fundamentals of Nursing*.

[26] Son C. H. (2018). The effect of ethical climate on the moral distress in emergency department nurses.

[27] Akdeniz M., Yardımcı B., Kavukcu E. (2021). Ethical considerations at the end-of-life care. *SAGE Open Medicine*.

[28] Choi Y. J. (2018). The influence factor of nurses’ terminal care attitude.

[29] Hwang S. H. (2018). The influence of nurses’ spirituality and awareness of death on the attitudes toward care of the dying.

[30] Han H. S., Choe W. S. (2008). Role accomplishment and job satisfaction of hospice nurse. *Korean Journal of Hospice Care*.

[31] Son Y. J., Park J. S. (2021). Effects of perception of death, terminal care stress, and resilience on the terminal care performance of clinical nurses. *Journal of East-West Nursing Research*.

[32] McCourt R., Power J. J., Glackin M. (2013). General nurses’ experiences of end-of-life care in the acute hospital setting: a literature review. *International Journal of Palliative Nursing*.

[33] Cho E. A., Ki J. S. (2021). Effects of perception of good death and knowledge toward advance directive on attitude toward withdrawal of life-sustaining treatment among university hospital nurses. *The Journal of the Korea Contents Association*.

